RETRACTED

# Spatial distribution of elements, environmental effects, and economic potential of waste from the Aksu ferroalloy plant [Kazakhstan]

**DOI:** 10.1371/journal.pone.0283251

**Published:** 2023-04-19

**Authors:** Ruslan Safarov, Zharas Berdenov, Raushan Urlibay, Yuriy Nossenko, Zhanat Shomanova, Zhuldyz Bexeitova, Andrej Kulak, Imre Varga, Andrej Balog, Rita Nyizsalovszki Domjánné, Lóránt Dénes Dávid

**Affiliations:** 1 Faculty of Natural Sciences, Chemistry Department, L.N. Gumilyov Eurasian National University, Nur-Sultan, Kazakhstan; 2 Faculty of Natural Sciences, Department of Physical and Economic Geography, L.N. Gumilyov Eurasian National University, Nur-Sultan, Kazakhstan; 3 Environment and Chemical Technologies Department, Innovative University of Eurasia, Pavlodar, Kazakhstan; 4 High School of Nature Science, Pavlodar Pedagogical University, Pavlodar, Kazakhstan; 5 Eurasian Center for Innovative Development, Nur-Sultan, Kazakhstan; 6 Faculties of Humanities and Social Sciences, Department of Physical Education and Sport, Toraighyrov University, Pavlodar, Kazakhstan; 7 Faculty of Social Sciences, Savaria Department of Business Economics, Institute of Economics, Eötvös Loránd University, Szombathely, Hungary; 8 Institute of Rural Development and Sustainable Economy, Hungarian University of Agriculture and Life Sciences [MATE], Gödöllő, Hungary; 9 Institute of Economics and Social Sciences, Eszterházy Károly Catholic University, Eger, Hungary; 10 Faculty of Economics and Business, John von Neumann University, Kecskemét, Hungary; Szechenyi Istvan University: Szechenyi Istvan Egyetem, HUNGARY

## Abstract

The utilization or secondary use of technogenic waste is a relevant problem for the current economy. To assess the environmental influence and economic potential, it is necessary to study the elemental content of technogenic objects and to reveal the tendencies of the spatial distribution of elements, components, and indices such as the pollution coefficient. In this study, we performed elemental analysis, and calculation of indicators: average gross content, hazard quotients, concentration coefficients of metals, and total pollution coefficients of ground samples taken from the ash-slag storage of the Aksu ferroalloy plant [Aksu, Pavlodar region, Kazakhstan]. Maps of the spatial distribution of concentrations of elements and total pollution coefficients were created. The territory of the studied ash-slag storage by the level of soil contamination should be considered as an environmental disaster zone. The given statistical data on the number of oncological and respiratory diseases indirectly indicated the negative influence of open storage of ash-slag waste. The studied ground was of chromium-manganese geochemical specialization. The calculated volume of the accumulated waste mass by the approximating method was 1 054 638.0 m^3^. The calculated approximate weight of the accumulated waste was 23 679 576.0864 tons, including 1 822 972.2 tons of chromium, 1 727 354.0 tons of manganese, and 953 813.3 tons of iron. The large amounts of valuable components retained in the waste mass led us to conclude that the studied technogenic object can be considered as a secondary field to produce various technological products. Moreover, valuable metals can be extracted as metal concentrates.

RETRACTED

## Introduction

According to the current data, metallurgy is one of the leading sectors in Kazakhstan’s economy [1–3]. Its share was 21.2% of the total volume of industrial production [processing and mining] in 2020 [3–5]. The metallurgy industry is located mainly in three regions of Kazakhstan: Karaganda, East Kazakhstan, and Pavlodar [3,4,6]. As of April 1^st,^ 2021, there were 391 metallurgical companies in Kazakhstan, including 29 large, 29 medium, and 333 small companies [7]. The main metallurgy companies of Kazakhstan are Kazakhmys Corporation LLP, KazZinc LLP, Aluminum of Kazakhstan JSC, Kazakhstan Electrolysis Plant JSC, Ust-Kamenogorsk Titanium and Magnesium Combine JSC in nonferrous metallurgy, JSC "ArcelorMittal Temirtau", TNK "Kazchrome" [including Aksu ferroalloy plant], Zhayremsky mining and processing plant, Sokolovsko-Sarbayskoye Mining and Production Association, JSC "Temirtau Electrometallurgical Combine", Casting LLP, and others in ferrous metallurgy [1,2,5].

The main exported metallurgical products of Kazakhstan are as follows: ferrochromium; copper ores and concentrates, iron ores and concentrates, and untreated, unalloyed zinc [1,5,7]. However, despite the rich mineral resources in Kazakhstan, the metallurgical branch mainly has a raw material orientation [7]. The absence of sufficient processing in metallurgy is the main constraint in the development of high-tech national economic sectors, such as machinery, transportation, and construction branches [3,8]. Meanwhile, the weak development of machinery and transportation negatively affects the competitiveness of the oil refining, chemical, woodworking, construction, and agriculture industries [5]. The raw material orientation in metallurgy in Kazakhstan is one of the main risks affecting this industry [3]. Should there be a reduction in the global demand for metals, Kazakhstan would suffer from the lack of technological advantages compensating the reduction in the production rates.

It is commonly known that the main sources of soil contamination are industrial and energy enterprises, household waste, and vehicles [9–11]. Over 22 billion tons of waste, including approximately 4 billion tons of mining waste, over 1.1 billion tons of toxic waste, and 105 million tons of metallurgical processing waste have accumulated as a result of the activities of nonferrous metallurgy enterprises [12]. Interestingly, in Kazakhstan no more than 2% of accumulating waste is processed and utilized nowadays [3,13].

RETRACTED

The area occupied by nonferrous metallurgical waste storage amounts to approximately 15 thousand hectares, of which rock dumps occupy 8 thousand, tailings of processing plants occupy approximately 6 thousand, and dumps of metallurgical plants occupy more than 500 hectares [12]. Alarmingly, looking at the volumes of waste produced in the ferrous metallurgy and chemical industries, data predicts the same growth rates for these industries. Pollutants migrate into the environment as a result of the constant increase in the volume of accumulated waste owing to the unsettled places of their storage and disposal [10,14].

The Aksu ferroalloy plant [AFP] belongs to the Joint-Stock Company «Transnational Company "Kazchrome"», which is part of the Eurasian Resources Group [ERG]. It is one of the largest metallurgical enterprises in the world for the production of chromium, siliceous, and manganese alloys [15]. The plant is located in Aksu, Pavlodar region, Kazakhstan. The capacity of AFP is more than 1 million tons of ferroalloys per year. The plant consists of four main production workshops and 26 electric furnaces and also includes a slag processing complex [16]. The main products of this plant are high-carbon ferrochromium, ferrosilicochrome, ferrosilicomanganese, and ferrosilicon [17]. The product grades and waste types are listed in **Table 1**.

**Table 1:** Main products and waste of the Aksu ferroalloy plant [18].

Products	Content, wt. %						
	Cr	Mn	Fe	Si	C	P	S
**HCFeCr**	69–70		balance	0.5	7.8–9.2	0.02–0.03	0.02–0.04
**FeSiCr**	31–36		balance	43–49	0.04–0.05	0.025	0.02
**SiMn**		66–67	balance	16–17	1.5–2.0	0.13–0.15	0.02
**FeSi75**				75			
**Waste**	Cr_2_O_3_	MnO					
**HCFeCr slag**	4.0–5.3						
**FeSiMn slag**		11.1–13					

**Table 1** shows the significant contents of Cr- and Mn-containing components. Additionally, Fe components are assumed to be present in the waste. The detailed elemental content of ferroalloy production waste is a subject of research because of the opportunities for reuse or deep processing of the material to obtain valuable products. Production waste is stored mainly in the ash-slag storage of AFP.

The secondary use of deposited waste mass is a relevant issue [19–21]. To solve this problem, it is necessary to study technogenic objects from environmental and economic points of view. To assess the ecological impact, it is necessary to assess environmental indices, such as the total pollution coefficient, and define the gross amounts of the valuable waste components [22]. The study focuses on the most relevant waste elements, including Cr, Mn, and Fe. The study of the spatial distribution of elements provides an estimate of the total volume and weight of the deposited waste, which is necessary to assess the gross amounts of the target components. However, there are no recent studies on the described information for ash-slag storage of AFP.

RETRACTED

Our study aims to reveal the elemental content of ground samples taken from different locations of the ash-slag storage of AFP, study also attempts to find an automatic method for finding the distribution of the elements in the production waste, and, finally, the study wants to assess environmental risks and economic potential by calculating the average elemental content, as well as the total pollution coefficient [23–26], calculating the approximate volume of the waste remaining in the storage, calculating the approximate amounts of the element reserves deposited in the studied technogenic object.

## Methods

### Study area

The object of this research is the ash-slag storage of the Aksu ferroalloy plant [Aksu, Kazakhstan]. The storage area is oval, with an area of ~203 073 m^2^ [**Fig 1**]. The waste was partially covered by water. In many locations, the waste level was higher than the water level.

**Fig 1:** Sampling map of ash slug storage at the Aksu Ferroalloy Plant [Aksu, Kazakhstan]. Coordinate system: WGS 84: Pseudo-Mercator EPSG: 3857, satellite map: ESRI Satellite [ArcGIS/World_Imagery], scale: 1:5827.

### Sampling

Fifty samples with a ground weight of at least 200 g were sampled from a layer of approximately 50 cm under the top ground surface. Sampling was performed using plastic equipment, and a sampling map is shown in **Fig 1**. The distance between the sample points was not less than 100 m. The samples were transported and stored in plastic containers for preservation from direct sunbeams. Before the analyses, the waste samples were air-dried.

### Elemental analysis

The elemental contents of the samples were analyzed using an X-ray fluorescent analyzer BRA-18 [Russia]. The analyzer can detect the contents of chemical elements from Na to U in solid, powder, and liquid samples [27]. The method uses the measurement of the wavelength and intensity of fluorescent radiation [X-ray] from the excited atoms of the sample [28].

## Results and discussion

### Elemental analysis

The results of the elemental analysis correlated with the production of AFP. Mn-, Fe-, and Cr-containing alloys have the main weight share in the samples since they are the plant’s main products, the maximum Cr content was 8.5406 wt. %, Mn was 7.4498 wt.%, and Fe was 5.8937 wt. % [**Table 2**]. Overall, the results show that the Ca content is not higher than 2.35%, Ti varies in the range of 0.7–0.95%, and the contents of V, Co, Ni, and Cu are even and are approximately 0.02, 0.006, 0.015, and 0.006 wt. %, respectively. The largest amount of Zn was 0.1194 wt. % and Pb was 0.0080 wt.%. Thus, the high content of valuable transition metals Cr, Mn, and Fe provides opportunities to use the waste material from the ash-slag storage of AFP to obtain new products or as a raw material in the deep extraction of these metals.

RETRACTED

**Table 2:** Elemental content [wt.%] of ground samples from ash-slag storage of Aksu ferroalloy plant.

Sample ID	Cl	Сa	Ti	V	Mn	Fe	Co	Ni	Сu	Zn	Pb	Cr	Sum	Other
**1**	0.0036	2.1080	0.8836	0.0220	7.2898	3.8628	0.0054	0.0129	0.0055	0.0777	0.0040	7.9493	22.2246	77.7754
**2**	0.0036	1.4367	0.8073	0.0211	7.4482	5.8931	0.0054	0.0138	0.0056	0.1161	0.0078	8.5405	24.2992	75.7008
**3**	0.0035	1.7721	0.8361	0.0209	7.3060	4.2964	0.0055	0.0147	0.0057	0.0981	0.0059	8.1408	22.5056	77.4944
**4**	0.0036	2.1114	0.8846	0.0226	7.2911	3.8638	0.0054	0.0132	0.0059	0.0779	0.0041	7.9559	22.2394	77.7606
**5**	0.0037	1.4500	0.8240	0.0228	7.4492	5.8926	0.0054	0.0148	0.0052	0.1194	0.0079	8.5406	24.3356	75.6644
**6**	0.0035	1.7755	0.8527	0.0216	7.3103	4.3030	0.0053	0.0157	0.0064	0.0981	0.0057	8.1439	22.5416	77.4584
**7**	0.0035	1.7755	0.8384	0.0222	7.3093	4.2957	0.0061	0.0157	0.0064	0.0977	0.0059	8.1542	22.5306	77.4694
**8**	0.0034	2.1097	0.8846	0.0230	7.3098	3.8638	0.0057	0.0129	0.0055	0.0779	0.0041	7.9496	22.2499	77.7501
**9**	0.0035	1.4400	0.8076	0.0224	7.4488	5.8937	0.0056	0.0140	0.0056	0.1163	0.0079	8.5372	24.3028	75.6972
**10**	0.0034	1.7711	0.8394	0.0212	7.3070	4.2957	0.0052	0.0148	0.0056	0.0981	0.0059	8.1397	22.5072	77.4928
**11**	0.0035	2.1087	0.8736	0.0226	7.2897	3.8614	0.0055	0.0127	0.0054	0.0780	0.0041	7.9593	22.2245	77.7755
**12**	0.0036	1.4400	0.8206	0.0214	7.4488	5.8934	0.0064	0.0139	0.0056	0.1158	0.0080	8.5406	24.3182	75.6818
**13**	0.0034	1.7755	0.8377	0.0222	7.3160	4.2974	0.0058	0.0148	0.0057	0.0987	0.0059	8.1275	22.5106	77.4894
**14**	0.0034	2.1080	0.8836	0.0236	7.2915	3.8626	0.0059	0.0142	0.0054	0.0778	0.0039	7.9426	22.2226	77.7774
**15**	0.0037	1.4370	0.8080	0.0218	7.4475	5.8921	0.0059	0.0145	0.0056	0.1154	0.0078	8.4412	24.2003	75.7997
**16**	0.0034	1.7738	0.8371	0.0219	7.3126	4.2974	0.0058	0.0153	0.0056	0.0982	0.0059	8.1410	22.5181	77.4819
**17**	0.0035	1.7711	0.8394	0.0229	7.3073	4.2974	0.0069	0.0143	0.0058	0.0977	0.0057	8.1375	22.5096	77.4904
**18**	0.0034	2.1094	0.8837	0.0221	7.2897	3.8641	0.0057	0.0125	0.0054	0.0780	0.0039	7.9359	22.2138	77.7862
**19**	0.0036	1.4369	0.8006	0.0224	7.4495	5.8924	0.0058	0.0139	0.0055	0.1164	0.0080	8.5072	24.2622	75.7378
**20**	0.0035	1.7755	0.8227	0.0210	7.3160	4.2897	0.0059	0.0148	0.0056	0.0985	0.0060	8.1338	22.4930	77.5070
**21**	0.0035	1.7655	0.8227	0.0208	7.3056	4.2764	0.0043	0.0145	0.0056	0.0984	0.0057	8.1275	22.4505	77.5495
**22**	0.0034	1.7621	0.8244	0.0212	7.3026	4.3030	0.0043	0.0147	0.0055	0.0980	0.0059	8.1292	22.4745	77.5255
**23**	0.0034	2.1087	0.8769	0.0223	7.2831	3.8761	0.0051	0.0130	0.0054	0.0764	0.0039	7.9526	22.2270	77.7730
**24**	0.0036	1.4300	0.8074	0.0228	7.4498	5.8897	0.0064	0.0139	0.0055	0.1141	0.0080	8.4405	24.1918	75.8082
**25**	0.0035	1.7711	0.8327	0.0216	7.3080	4.2964	0.0057	0.0148	0.0056	0.0982	0.0057	8.1295	22.4929	77.5071
**26**	0.0036	2.3250	0.8205	0.0225	7.4279	4.2932	0.0052	0.0198	0.0055	0.0141	0.0012	7.8432	22.7816	77.2184
**27**	0.0036	1.9039	0.9590	0.0219	7.2533	3.4403	0.0052	0.0140	0.0055	0.0141	0.0011	6.9497	20.5715	79.4285
**28**	0.0036	1.9587	0.8764	0.0214	7.2560	3.4951	0.0051	0.0167	0.0055	0.0141	0.0011	7.4206	21.0744	78.9256
**29**	0.0036	1.4654	0.8101	0.0212	7.0358	2.5949	0.0050	0.0108	0.0054	0.0122	0.0010	6.4620	18.4274	81.5726
**30**	0.0036	1.8635	0.9060	0.0225	7.1715	3.1814	0.0051	0.0170	0.0055	0.0138	0.0011	7.1891	20.3799	79.6201
**31**	0.0037	1.9778	0.7752	0.0222	7.3455	3.6106	0.0050	0.0158	0.0054	0.0139	0.0010	7.4370	21.2131	78.7869
**32**	0.0035	2.3317	0.8272	0.0248	7.4379	4.2934	0.0064	0.0200	0.0053	0.0140	0.0011	7.7765	22.7417	77.2583
**33**	0.0035	1.9026	0.9490	0.0235	7.2531	3.4370	0.0053	0.0146	0.0053	0.0139	0.0010	6.8830	20.4920	79.5080
**34**	0.0034	1.9604	0.8750	0.0216	7.2520	3.4974	0.0048	0.0169	0.0053	0.0143	0.0011	7.4240	21.0763	78.9237
**35**	0.0036	1.4721	0.8087	0.0213	7.0360	2.5849	0.0054	0.0112	0.0053	0.0121	0.0010	6.3953	18.3570	81.6430
**36**	0.0034	1.8701	0.8860	0.0223	7.1848	3.1914	0.0053	0.0157	0.0053	0.0140	0.0012	7.1861	20.3856	79.6144
**37**	0.0035	1.9779	0.7768	0.0223	7.3457	3.6140	0.0053	0.0162	0.0053	0.0136	0.0037	7.4377	21.2218	78.7782
**38**	0.0035	2.3283	0.8189	0.0227	7.4292	4.2798	0.0055	0.0197	0.0055	0.0154	0.0012	7.8435	22.7732	77.2268
**39**	0.0036	1.9026	0.9593	0.0242	7.2526	3.4420	0.0054	0.0146	0.0056	0.0144	0.0010	6.9504	20.5757	79.4243
**40**	0.0035	1.9611	0.8754	0.0216	7.2460	3.4984	0.0055	0.0169	0.0056	0.0141	0.0011	7.4205	21.0697	78.9303
**41**	0.0034	1.4661	0.8334	0.0213	7.0425	2.5955	0.0052	0.0115	0.0053	0.0123	0.0010	6.4653	18.4630	81.5370
**42**	0.0036	1.8641	0.9076	0.0225	7.1725	3.1814	0.0055	0.0180	0.0054	0.0139	0.0011	7.1865	20.3820	79.6180
**43**	0.0035	1.9761	0.7748	0.0232	7.3457	3.6107	0.0054	0.0152	0.0053	0.0138	0.0010	7.4037	21.1784	78.8216
**44**	0.0036	2.3223	0.7872	0.0226	7.4305	4.2598	0.0056	0.0197	0.0055	0.0134	0.0010	7.7765	22.6478	77.3522
**45**	0.0035	1.8906	0.9457	0.0215	7.2529	3.4170	0.0055	0.0126	0.0053	0.0139	0.0012	6.9330	20.5028	79.4972
**46**	0.0036	1.9421	0.8734	0.0213	7.2227	3.4618	0.0055	0.0151	0.0056	0.0143	0.0010	7.4173	20.9835	79.0165
**47**	0.0035	1.4488	0.8067	0.0239	7.0352	2.5882	0.0051	0.0107	0.0053	0.0123	0.0010	6.3953	18.3359	81.6641
**48**	0.0035	1.8401	0.8926	0.0223	7.1448	3.1880	0.0053	0.0168	0.0055	0.0135	0.0009	7.1861	20.3194	79.6806
**49**	0.0037	1.9444	0.7885	0.0228	7.3322	3.6040	0.0053	0.0145	0.0052	0.0138	0.0010	7.4373	21.1726	78.8274
**50**	0.0036	1.9454	0.8430	0.0211	7.2460	3.4934	0.0054	0.0154	0.0051	0.0140	0.0011	7.4106	21.0041	78.9959

According to the value of the average gross content, the studied elements were arranged in the following descending order: Cr > Mn > Fe > Сa > Ti > Zn > V > Ni > Co > Сu > Cl > Pb. The coefficient of variation of the average gross contents of the studied elements ranged from 0.0035 wt. % [Pb, Cl] to 7.6986 wt.% [Cr]. The variation in the absolute gross metal content was higher, ranging from 0.0034 [Pb] to 8.5406 [Cr].

RETRACTED

### Environmental assessment

Logically, keeping the waste mass in storage leads to the alienation of natural territory. When studying the environmental aspects of technogenic objects, it is necessary to determine the degree of effect on human health, the use of green solutions and the potential for tourism development [29–32]. Two obvious assessment methods are to determine the average excess concentration of heavy metals over the level of maximum permissible concentrations [MPC] in the ground and to calculate the total pollution coefficient Zc [23–26].

Analysis in comparison with MPC [**Table 3**] showed that all waste samples exceeded the declared levels of MPC in Kazakhstan based on the heavy metal content.

**Table 3:** Assessment of gross content of heavy metals in waste samples regarding maximum permissible concentrations [MPC] [n = 50].

Metal	Average gross content, mg/kg	Range of gross content [Lim], mg/kg	Variation Coefficient, %	MPC, mg/kg	Average HQ	Share of samples where HQ > 1, %
**Cu**	55.08	51–64	4	33	1.67	100
**Fe**	40280.74	25849–58937	22	-	-	-
**Zn**	556.02	121–1194	78	23	24.17	100
**Pb**	35.36	9–80	75	32	1.10	52
**Mn**	72947.90	70352–74498	2	1500	48.63	100
**V**	221.78	208–248	4	150	1.48	100
**Co**	54.74	43–69	9	5	10.95	100
**Ni**	148.74	107–200	14	4	37.18	100
**Cr**	76985.56	63953–85406	8	6	12830.93	100

The excess value was expressed by hazard quotients [HQ] [33–35], where HQ = actual gross content [mg/kg]/MPC [mg/kg]. The HQ levels were extremely high and achieve 12 830 times in the case of chromium. Only in the case of lead was the share of samples exceeding the MPC lower than 100% and reached 52%.

RETRACTED

The characteristics of technogenesis can be seen in comparison with versatile international indices, such as MPC by Kloke and Clarke in the soil and Clarke in the lithosphere [**Table 4**]. In the ground samples, the Zn content exceeded the MPC by Kloke by 1.85 times, soil Clarke by 3.52 times, and lithosphere Clarke by 6.7 times. The Mn content exceeded that of soil Clarke 100 times, and that of lithosphere Clarke 72.95 times. The Cr content exceeded the MPC by 769.86 times, soil Clarke by 962.32 times, and lithosphere Clarke by 927.54 times.

**Table 4:** Values of the average gross content of heavy metals in waste samples in comparison with conventional indicators.

Metal	Average gross content, mg/kg	MPC by Kloke, mg/kg [36]	Clarke in soil, mg/kg [37]	Clarke of the earth’s crust, mg/kg by P. Vinogradov [1962] [38]	Background, mg/kg	Kc
**Cu**	55.08	100	39	47	17.9	3.08
**Fe**	40280.74	-	22300	46500	19274	2.09
**Zn**	556.02	300	158	83	42.4	13.11
**Pb**	35.36	100	54.5	16	15.7	2.25
**Mn**	72947.9	-	729	1000	525.8	138.74
**V**	221.78	50	104.9	90	47.8	4.64
**Co**	54.74	50	14.1	18	7.2	7.6
**Ni**	148.74	50	33	58	28.8	5.16
**Cr**	76985.56	100	80	83	36.9	2086.33

The summary indicator of pollution [Zc] is calculated as the sum of excess coefficients of concentrations of chemical elements accumulating in technogenic anomalies and is calculated using the formula of the Saeta index [26].

$$Z_{c}=\sum_{i}{Kc}_{i}-[n-1]$$

where Kc is the concentration coefficient of the substance and n is the number of analyzed contaminant elements with Kc > 1. Kc was calculated using the following formula:

$$Kc=\frac{C}{C_{0}}$$

where C is the content of the contaminant element at a given point, and C_0_ is the content of the contaminant element in the background soil. Background samples were taken 80 km from the object in a pollution-free territory.

In the formulas for geochemical specialization [39,40], the numerical index attached to the symbol of the chemical element refers to the multiplicity of the average values of the concentration coefficients [Kc] for the entire set of points included in the contour of the object [39]. The formula for geochemical specialization [41] of ground samples from the ash-slag storage of AFP is Cr_2086.33_Mn_138.74_Zn_13.11_Co_7.6_Ni_5.16_V_4.64_Cu_3.08_Pb_2.25_Fe_2.09_. On average, the studied ground is of chromium-manganese geochemical specialization.

RETRACTED

The assessment of the danger of soil contamination by a complex of pollutant elements according to indicator Zc was carried out on an evaluation scale. Gradations of the assessment scale were developed based on the study of indicators of the health status of the population living in territories with different levels of pollution. The calculated average Zc for the ground ash slag storage of the AFP was 2 253. According to the criteria for assessing the environmental situation of territories to identify an environmental emergency and environmental disaster zone, 1 992 areas with Zc more than 128 are characterized by very high soil contamination and should be considered environmental disaster zones.

Zc values were calculated for every sample to create a 3D map of the Zc distribution in the studied territory [**Fig 2**]. Analysis of the distribution of geochemical indicators obtained from the results of ground sampling on a regular grid provides the spatial structure of pollution.

**Fig 2:** 3D spatial distribution of Zc levels on the ash-slag storage of AFP. Coordinate system: WGS 84: Pseudo-Mercator EPSG:3857.

Zc spatial data were overlapped as layers on the map using GIS technology. Data visualization was performed using interpolation by inverse distance weighting [IDW] in QGIS Software [v. 3.24.2-Tisler]. The radius of influence of each of the starting points on the interpolated variable is determined by the value of "weights" [**Fig 3**].

**Fig 3:** 2D spatial distribution of Zc levels on the ash-slag storage of AFP. Coordinate system: WGS 84: Pseudo-Mercator EPSG: 3857, satellite map: ESRI Satellite [ArcGIS/World_Imagery], scale: 1:5827, method of interpolation: QGIS IDW, distance coefficient = 5.0, pixel size = 0.275182.

In addition, a complex layer map was created to demonstrate the distribution characteristics of the detected elements [**Figs 4 and 5**].

**Fig 4:** Spatial distribution of Pb on the ash-slag storage of AFP. Coordinate system: WGS 84: Pseudo-Mercator EPSG: 3857, satellite map: ESRI Satellite [ArcGIS/World_Imagery], scale: 1:5827, method of interpolation: QGIS IDW, distance coefficient = 5.0, pixel size = 0.275182.

**Fig 5:** Spatial distribution of Zn on the ash-slag storage of AFP. Coordinate system: WGS 84: Pseudo-Mercator EPSG: 3857, satellite map: ESRI Satellite [ArcGIS/World_Imagery], scale: 1:5827, method of interpolation: QGIS IDW, distance coefficient = 5.0, pixel size = 0.275182.

When analyzing the spatial distribution of metals, it is necessary to consider variation coefficients to assess the degree of uniformity in the dissemination of elements [42,43]. The variation coefficient allows us to compare the uniformity of the values, even with different scales of data. The variation coefficient [%] is calculated by the formula [43]: c = D · 100/x͞, where D is the standard deviation and x͞ is the medium value.

RETRACTED

In statistics, it is accepted that if the value of the coefficient of variation is less than 33%, then the set is considered uniform; otherwise, it is random [33–64%] or cluster distributed [>64%] [44]. In general, the coefficient of variation is used to estimate the relative spread of the data in the sample. Therefore, the colors on the maps represent the relative concentration dispersion divided into eight equal classes. The classifications for each element are shown in the corresponding maps.

The analysis showed that the value of the variation coefficient for the Zc index was 8%, which indicates the uniformity of the index. This is natural because of the technogenic nature of the genesis of the studied ground. Waste is produced by a steady process over many years. Meanwhile, visual analysis of the map shows that the value of Zc in the northwest part of the ash-slag storage is higher. This can be explained by the fact that the output of the cleaning system is placed in that part of the storage; the mass of the waste is then disseminated to other parts of the storage.

Considering elemental dissemination, we can see that Zn and Pb have cluster [mosaic] distribution characteristics. **Figs 4 and 5** show a mosaic picture of the distribution of these metals in the ash slag storage area. Both metals were detected in the northwestern part of the storage area, and their concentrations significantly decreased in the southeastern direction. Considering the variation coefficients, other metals were disseminated more or less uniformly, but the relative content was higher in the northwestern part.

### Statistics on the health issues

The environmental effects of heavy metals migration can be revealed through accumulation in biomass, soil, and groundwater. Heavy metals finally migrate in living organisms and at reaching the exceeding amount they can change the structure of proteins and nucleic acids, negatively influence metabolism, disturb the structure and permeability of cell membranes, and cause violations of the work of internal organs. The main and most dangerous group of human diseases caused by heavy metals is oncology.

According to the data from the statistical digest of the Ministry of Health of the Republic of Kazakhstan for 2020 [45], the number of oncology disease cases number in the Pavlodar region increased from 1111.1 to 1265.7 cases per 100 thousand living people. The number of oncology diseases in the Pavlodar region is growing. Thus, in 2019 the Pavlodar region was in 4^th^ place, and in 2020 it moved to 1^st^ place by this indicator [**Fig 6**].

RETRACTED

**Fig 6:** Number of oncology disease cases per 100 thousand living people in regions and cities of regional significance in Kazakhstan [45].

Migration of elements-pollutants mainly goes by air. Dust particles of pollutants can attack the human respiratory system. According to human health statistics [45,46], the Pavlodar region is a leading region in the number of cases of respiratory diseases. The Pavlodar region takes 1^st^ place in this group of diseases in both the 2019 and 2020 years [**Fig 7**].

**Fig 7:** Number of respiratory disease cases per 100 thousand living people in regions and cities of regional significance in Kazakhstan [45].

The aim of the research was not to reveal the direct relations between the ash-slag dump and the health indicators of people living in the region. However, at first glance, it is obvious, that influence of such large enterprises as AFP [Aksu city] and the Pavlodar aluminum plant [Pavlodar city], causes a significant increase in the number of oncological and respiratory diseases cases in the Pavlodar region. The influence of pollution from the studied technogenic object can be decreased using proper means of protection and preventative measures. From the other point of view utilization of the waste leads to the disappearance of the issue origin. To understand the amount of valuable components going for utilization, it is necessary to carry out the technogenic resource assessment.

### Technogenic resource assessment

Knowing the elemental content, it is possible to calculate the storage ability of valuable raw materials as a secondary field. First, the total weight of waste deposited in the storage must be calculated. The total weight could not be calculated precisely, which is why we used the approximated value. The approximate total weight was calculated using the following formula: m = ρ · V, where ρ is the bulk density [kg/m^3^], and V is the volume [m^3^].

A bowl-shaped model of the bottom surface geometry was used to calculate the volume of waste deposited in the studied storage. The storage was an industrial facility that involves excavation with an approximate bowl form. The maximum depth is at the center of the excavation and reaches 4 m.

For each point, the relative distance [Lr] from the nearest zero point at the edge of the reservoir to the given point was determined. The distance was relative because regardless of the location of a given point, the maximum distance to the nearest zero point was assumed to be 1.0 and corresponded to the shortest distance from the point of greatest depth to that zero point along a straight or broken line with the intersection of a given point [**Fig 8**].

RETRACTED

**Fig 8:** Contour of an excavation with marked zero points [on the edge] and the point of the greatest depth [point D].

The relative distance [L_r_] was calculated as:

$$L_{r}=\frac{L[OX]}{L(OX)+L[XD]}$$

where L[OX] is the absolute distance from the nearest zero point to point *i* [m], and L[XD] is the absolute distance from the point of the greatest depth to point *i* [m] [**Fig 8**].

The absolute distances were calculated by knowing the coordinates of points in the coordinate system WGS 84: Pseudo-Mercator EPSG:3857, which allowed us to obtain coordinates in meters. The values of the X and Y coordinates were obtained using GIS [QGIS software]. The method of calculating the absolute distance between two points on a plane is typically reduced to solving a triangle, or, in other words, finding its hypotenuse. The Pythagorean theorem is used for this purpose. The formula for determining the distance between points A[Xa, Ya] and B[Xb, Yb] on the plane is as follows:

$$d=\sqrt{{\left(X_{b}-X_{a}\right)}^{2}+{\left(Y_{b}-Y_{a}\right)}^{2}}$$

where Xa and Ya are the coordinates of the first point A and Xb and Yb are the coordinates of the second point B.

By modeling the bowl-shaped curve of the bottom surface, we constructed a curve of the dependence of the depth value on the relative distance to the nearest zero point [Lr]. Using MS Excel tools, we built a trend line and derived its formula with coefficients [**Fig 9**]. For a bowl-shaped bottom, the logarithmic curve most closely describes the geometry.

**Fig 9:** The curve of the dependence of the depth on the relative distance from the nearest zero point [Lr].

The resulting formula is y = 1.3898ln[x] + 4.158, which allows the calculation of depth [y] based on the relative distance from the nearest zero point [x].

To calculate the storage volume, points were placed on a uniform grid with steps of 10 m. In total, 5 364 points were taken in the area of the studied ash slag storage. Points were obtained using GIS with the coordinate system WGS 84: Pseudo-Mercator EPSG:3857, which allows the coordinates to be obtained in meters. Depth values were calculated for each point. Thus, using the cuboid volume formula, the volumes of every cuboid with a width of 10 m, length of 10 m, and height [depth] were calculated. The formula used was V_i_ = a^2^ · h, where a is the grid step [m] and h is the excavation depth at a given point [m].

The sum of the obtained cuboid volumes provides the required total volume of waste mass deposited on storage. The obtained volume was 1 054 638.0 m^3^. The average bulk density of the samples from the studied ash-slag storage was 22.4528 g/сm^3^ or 22 452.8 kg/m^3^. Thus, the total mass of the deposited waste is 1 054 638.0 · 22 452.8 = 23 679 576 086.4 kg or 23 679 576.0864 tons.

RETRACTED

Using the elemental content data, the approximate deposit of each detected element [in the elemental state] was calculated [**Table 5**]. Therefore, storage has great economic potential. The studied technogenic object can be considered a secondary field to produce various technological products, such as additives in building mixes, catalysts, and additives for steel production, and valuable metals can be extracted as metal concentrates.

**Table 5:** Assessment of gross content of heavy metals in waste samples regarding maximum permissible concentrations [MPC] [n = 50].

Metal	Average gross content, wt. %	Approximate content in the ash-slag storage, tons
**Cu**	0.0055	1 302.4
**Fe**	4.0280	953 813.3
**Zn**	0.0556	13 165.8
**Pb**	0.0035	828.8
**Mn**	7.2947	1 727 354.0
**V**	0.0221	5 233.2
**Co**	0.0054	1 278.7
**Ni**	0.0148	3 504.6
**Cr**	7.6985	1 822 972.2

## Conclusion

In this study, the elemental content of waste placed on the ash slag storage of the Aksu Ferroalloy Plant [Aksu, Kazakhstan] was sampled at different locations and analyzed. Maps of spatial concentration distributions were created for each metal. A summary indicator of pollution [Zc] was calculated for each point, and the data were placed on the map. An environmental assessment was conducted, and an assessment of the reserves of valuable components present in the waste was performed. The metals revealed in the waste were Cu, Fe, Zn, Pb, Mn, V, Co, Ni, and Cr. The studied ground was characterized by chromium-manganese geochemical specialization.

The studied technogenic object, the ash-slag storage of the Aksu ferroalloy plant, is a typical product of technogenesis. This can be considered from two perspectives: First, it negatively affects the environment as a technogenic object. The territory used for the placement of this facility was alienated. This territory is characterized as an environmental disaster zone based on the level of contamination with elemental pollutants. Storage of this type of waste can negatively affect the health of staff and people living in the nearest proximity areas. The analysis of official health statistics reveals that the influence of AFP [Aksu city] can contribute to a significant increase in the number of oncological and respiratory disease cases in the Pavlodar region. Proper storage conditions, such as sufficient coverage of the slag level by water, can decrease these negative effects. These conditions should be controlled regularly. The environmental impact of ferrochrome production can be effectively contained using existing techniques and processes, such as preventative measures [for example, furnace design and slag composition], treatment of Cr[VI] containing material [for example, chemical treatment], and protection of employees by issuing enhanced PPE and strictly enforcing its use.

RETRACTED

Second, it was revealed that the studied waste had great economic potential. It can be a valuable raw material and is involved in a new cycle of production. Significant amounts of valuable metals such as Mn, Cr, and Fe can be extracted as metal concentrates or used for direct recycling. This approach leads to the discovery of new ways to modify production schemes by including new co-productions using waste as a raw material. One of the most promising ways to utilize the studied types of waste is the production of construction and refractory mixtures, commercial crushed stone and sand, catalysts, and metal concentrates. The metal concentrates can be considered in the production scheme of the Aksu ferroalloy plant; the return share can reach 10%.

## Supporting information

S1 File (PDF)
